# FLG Is a Potential Biomarker of Prognosis and Immunotherapy in Skin Cutaneous Melanoma

This article has been retracted.

**DOI:** 10.1155/2022/5160748

**Published:** 2022-05-14

**Authors:** Shaobo Wu, Yuxia Liang, Qijuan Zang, Zixuan Xing, Pan Yin, Ruifang Sun, Bingling Dai

**Affiliations:** ^1^Health Science Center, Xi'an Jiaotong University, Shaanxi, Xi'an 710061, China; ^2^Department of Imaging, The First Affiliated Hospital of Xi'an Jiaotong University, Shaanxi, Xi'an 710061, China; ^3^Department of Pathology, School of Basic Medical Sciences, Xi'an Jiaotong University, Shaanxi, Xi'an 710061, China; ^4^School of Pharmacy, Health Science Center, Xi'an Jiaotong University, Shaanxi, Xi'an 710061, China

## Abstract

**Background:**

Skin cutaneous melanoma is one of most aggressive type of cancers worldwide. Therefore, the identification of SKCM biomarkers is of great importance. FLG gene is one of the genes that encode proteins involved in epidermal formation. This was the first time to study the role of FLG in the prognosis and immune infiltrates of skin cutaneous melanoma.

**Methods:**

We downloaded the somatic mutation data of 471 SKCM patients from the Cancer Genome Atlas (TCGA) database and analyzed the mutation profiles with “MafTools” package. The expression of FLG and the overall survival in SKCM were analyzed by GEPIA. Additionally, univariate and multivariate Cox analyses were used to compare several clinical features with survival rates. We used TIMER to investigate FLG expression and collection of immune infiltration levels in SKCM, as well as cumulative survival in SKCM. Meanwhile, we also used CIBERSORT to investigate the association between FLG and cancer immune infiltration. In addition, gene set enrichment analysis (GSEA) was performed using the TCGA dataset. Furthermore, data from GEO and HPA was used to validate the results.

**Results:**

Single nucleotide polymorphism (SNP) happened more frequently than insertion or deletion, and C > T was the most common of SNV in SKCM. We selected the first 15 mutated genes by analyzing 471 melanoma samples, and the prognosis analysis showed that only the high expression of mutated FLG gene was significantly correlated with the poor prognosis of SKCM. Multivariate Cox analysis showed that age, the worse tumor status, less lymph node metastasis, and FLG expression were independent factors for prognosis. Specifically, lower infiltration levels of B cell, CD8+ T cells, neutrophils, and dendritic cells correlated with poor survival outcomes in SKCM. GSEA revealed that FLG is closely related to cancer pathways and epidermal cell proliferation. In addition, the previous conclusions can be verified from external data from GEO and HPA.

**Conclusion:**

The discovery of mutant gene FLG as a biomarker of SKCM helps elucidate how changes in the immune environment promote the occurrence of cutaneous melanoma. Further analysis suggested that FLG might be a new predictor of SKCM prognosis.

## 1. Introduction

Skin cutaneous melanoma (SKCM) is a major public health problem worldwide due to its extreme aggressiveness and dissemination; the mortality of SKCM patients is still increasing in many countries, and it causes 55 500 deaths annually [1]. At present, SKCM is usually diagnosed in the late grades of metastatic tumors, which could drive patients to a poor response to the therapeutic strategies [2]. Therefore, we need to explore potential biomarkers and therapeutic targets to improve the diagnosis and treatment of melanoma. Recently, numerous studies have shown that the dysfunction of immune system plays a key role in the progression of SKCM [3, 4]. The development of novel immunotherapies, such as anti-CTLA4 and anti-PD-1, has significantly improved melanoma patient outcomes [5, 6]. Therefore, immunotherapy is widely used in the treatment of melanoma. However, even immune checkpoint inhibitors (ICIs) such as antibodies targeting either the cytotoxic T-lymphocyte-associated protein 4 (CTLA-4) or the programmed death 1 (PD1) immune checkpoints, yet approximately 50% of the patients do not respond to treatment [7, 8]. Additionally, many studies had discovered that tumor mutation burden (TMB) was associated with immunotherapy in many cancer types [9, 10]. However, only one-fifth of cancer patients could benefit from immunotherapy [11]. Therefore, it is still necessary to find new immune-related therapeutic targets in SKCM.

The FLG gene is one of the genes that encode proteins involved in epidermal formation. Filaggrin is a structural, S100 calcium-binding epidermal SC protein [12]. The skin barrier function is largely dependent on SC. The interior of the corneocytes consists mainly of keratin filaments aggregated by FLG, which is one of components that provide a scaffold for the extracellular lipid matrix. Today, about 60 loss-of-function FLG mutations had been identified; the mutant spectrum was different among different populations [13]. There was a study found that skin sensitization, including the Th17 cell subpopulation, facilitated by acquired FLG defects or mutations can indirectly result in local but also systemic inflammation in distant organs [14, 15]. However, the role of FLG has not been explored in SKCM.

In this study, we firstly comprehensively analyzed the landscape of mutation profiles in SKCM samples from TCGA. Moreover, we investigated the FLG expression and correlation with the survival of SKCM patients and the relationship between FLG expression and the tumor-infiltrating immune cells in SKCM. The findings of this study helped us shed light on a potential correlation as well as a possible mechanism between FLG and tumor-immune interactions. Thus, FLG had the potential to become a novel predictor to evaluate prognosis and immune infiltration for SKCM patients.

## 2. Materials and Methods

### 2.1. Somatic Mutation Data Download and Preprocessing

Somatic cell mutation data were acquired from the Cancer Genome Atlas (TCGA) (https://tcga-data.nci.nih.gov/tcga/) [16]. From the data files of the four subtypes, the “Masked Somatic Mutation” data was selected and processed by the VarScan software. We prepared the variation annotation format (MAF) for somatic variation and used the “MafTools” R package, which provided multiple analysis modules to perform the visualization process. In addition, we downloaded gene expression profile and clinical information of SKCM patients, including 471 tumor samples and 1 normal sample. Subsequent processing excluded cases with insufficient or missing data on age, overall survival time, local invasion, lymph node metastasis, distant metastasis, and TNM stage. Finally, 322 cases with eligible clinical information were devoted into Cox regression analysis. Since all data in this study was from public databases, there was no ethical conflict that needed to be declared. We chose GSE15605 (normal = 16, tumor = 46) and GSE46517 (normal = 8, tumor = 31) as external data sets to confirm the expression level of FLG in normal and tumor tissues.

### 2.2. FLG Expression and Survival Analysis of SKCM

The analysis of FLG expression from TCGA database was conducted with the GEPIA website (http://gepia.cancer-pku.cn/). GEPIA is a public platform for analyzing the RNA sequencing expression data of 9,736 tumors and 8,587 normal samples from the TCGA and the GTEx projects [17]. We acquired samples from TCGA and used GEPIA to analyze the correlation between overall survival and FLG expression in SKCM. Meanwhile, a boxplot was drawn with disease state (tumor or normal) as the variable to show the differential expression of FLG in tumor and normal tissues. In addition, a boxplot of clinical staging with pathological staging as the variable was drawn to compare the expression of FLG in different pathological stages.

### 2.3. Immune Infiltrate Analysis

TIMER is a comprehensive resource for systematic analysis of immune infiltrates for diverse cancer types (https://cistrome.shinyapps.io/timer/) [18]. We evaluated FLG expression in SKCM and its correlation with the abundance of TIICs, including B cells, CD4^+^ T cells, CD4^+^ T cells, macrophages, neutrophils, and Dendritic cells by gene modules. Besides, we evaluated the mutation types of FLG with immune infiltrates in SKCM based on the “SCNA” module of TIMER. Boxplot was used to represent the distribution of each immune cell subpopulation in each SKCM mutant state, and two-side Wilcoxon rank sum test calculated *P* value was used to compare the differences of each immune cell subpopulation and normal infiltration level in each mutant state.

In addition, to assess the relative differences in gene expression in the sample set, we used an expression-based deconvolution algorithm called CIBERSORT (http://cibersort.stanford.edu/) [19]. Using CIBERSORT, we measured the immune response of 22 TIICs to assess their association with FLG expression in SKCM and to discover correlations between TIICs. *P* < 0.05 was considered statistically significant. Thus, we used 471 cutaneous melanoma samples from TCGA and divided them into half with low expression and half with high expression and then used to make a violin diagram. Moreover, to detect the correlation between 22 types of immune cells, we made the correlation heat map.

### 2.4. Gene Set Enrichment Analysis

Gene set enrichment analysis (GSEA) is commonly used to assess whether a particular gene set is significantly different in any two biological states. In this study, GSEA was used to analyze the differential signaling pathways of the activation of FLG low and high expression groups in SKCM patients. A sequence listing was subsequently generated based on the correlation of all genes with FLG expression, and it was performed 1000 times in this analysis. Thus, to be considered statistically significant, enrichment results had to satisfy two conditions: a false discovery rate (FDR) < 0.050 and a nominal *P* value < 0.050.

### 2.5. The Human Protein Atlas

The human protein atlas database (https://www.proteinatlas.org/) [20, 21] was used to analyze protein expression of FLG between normal and cutaneous melanoma tissues, which has both on mRNA and protein expression data on 44 different human tissues. The antibody-based protein profiling showed the protein expression level and location. Besides, its protein expression score is based on immunohistochemical data manually scored with regard to staining intensity (negative, weak, moderate, or strong) and fraction of stained cells (<25%, 25-75%, or >75%).

### 2.6. Statistical Analysis

All statistical analyses from TCGA were combined by the R software (version 3.6.3). To calculate the 95% CI and HR, we used both the univariate and multivariate models of the Cox analysis. Univariate survival analysis was used to compare several clinical factors with survival rate. Besides, multivariate Cox analysis was used to assess the influence of FLG expression and other pathological and clinical factors (age, gender, lymph node, distant metastasis, tumor status, and stage) on OS. *P* value < 0.05 was thought to be significant.

## 3. Results

### 3.1. Landscape of Mutation Profiles in SKCM

We downloaded the somatic mutation profiles of 471 SKCM patients from TCGA, including four types of data based on different processing software. We used the “MafTools” package to visualize the results of the VCF based mutation data. The mutation information for each gene in each sample was presented in the form of a waterfall map, with different colors representing different types of mutations and labeled at the bottom (Figure 1). Then, these mutations were further classified according to different classifications, among which missense mutation accounts for the majority (*y*-axis: variant classification; *x*-axis: number of samples) (Figure 2(a)), single nucleotide polymorphism (SNP) happened more frequently than insertion and deletion (Figure 2(b)), and C > T was the most common of single nucleotide variants (SNV) in SKCM (*y*-axis: SNV class; *x*-axis: proportion) (Figure 2(c)). In addition, we counted the number of changed bases in each sample and showed the mutation types in different colors in the boxplot of SKCM (Figures 2(d) and 2(e)). Thus, we showed the percentages of the top 10 mutated genes in SKCM (Figure 2(f)) and the coincidence and exclusion relationships between mutated genes (Figure 2(g)), where green represented cooccurrence and brown represented mutual exclusion.

### 3.2. Correlation between FLG Expression and Clinicopathological Features

We took the top 15 mutated genes for survival analysis by GEPIA and found the increased expression of FLG was significantly related to low overall survival (*P* = 0.0046) (Figure 3(b)). Besides, FLG expression was significantly lower in the SKCM compared to normal tissues (Log_2_FC < 1, *P* value < 0.01) (Figure 3(a)) and advanced pathological stage (*P* = 0.00205) (Figure 3(c)). As shown in Table 1, univariate analysis using Cox regression revealed that some factors, including age (HR = 1.02, *P* < 0.001), pathological stage (HR = 1.57, *P* < 0.001), and FLG expression (HR = 1.03, *P* < 0.001), were significantly associated with overall survival. In multivariate analysis (Table 1, Figure 3(d)) revealed that age, the worse tumor status, less lymph node metastasis, and FLG expression (*P* value = 0.020) were independent factors for prognosis.

### 3.3. Relationship between FLG Expression and Tumor-Infiltrating Immune Cells

To investigate whether the expression of FLG was associated with immune infiltration of SKCM, we assessed the correlation between FLG expression and the level of immune invasion by TIMER. Our results showed that FLG expression was associated with a better prognosis of SKCM. Lower infiltration levels of B cell, CD8^+^ T cells, neutrophils, and dendritic cells correlated with poor survival outcomes in SKCM (*P* < 0.05) (Figure 4(a)). We further evaluated the underlying relationships of the mutants of FLG with immune infiltrates in SKCM microenvironment. Compared with the immune infiltration levels in samples, diverse forms of mutation carried by FLG could commonly inhibit the immune infiltrates, including B cell, CD8+ T cell, CD4+ T cell, macrophage, neutrophil cell, and dendritic cell (Figure 4(b)). These results suggested that FLG plays a key role in SKCM immune infiltration. Additionally, our findings strongly support the significant role of FLG in immune infiltration. Moreover, we tried to ensure whether the tumor immune microenvironment was different in SKCM with high FLG levels compared to those with low levels. The 471 tumor samples were divided into 2 groups based on FLG expression. Then, we used CIBERSORT to explore gene expression profiles of downloaded samples to infer the density of 22 types of immune cells and applied its algorithm to the 22 immune cell subtypes helped assess differences in their expression levels in the high and low FLG expression groups. Results showed that B cell memory, macrophage M2, and mast cell resting were main immune cells effected by FLG expression (Figure 5(a)). Additionally, we assessed possible correlations between 22 types of immune cells (Figure 5(b)); the correlation heat map reflected a higher correlation within the proportions of different TIIC subgroups. Positive correlations were shown in red, whereas negative correlations were shown in blue. CD8+ T cells and macrophage M0 were negatively correlated (-0.65). By contrast, neutrophils and mast cells activated presented a significant positive correlation (0.78).

### 3.4. GSEA Investigation of FLG

We explored the potential biological functions of FLG through GO term and KEGG pathway analysis. As shown in Table 2, KEGG pathway analysis showed five pathways that had the strongest positive correlation with FLG expression, including small cell lung cancer, basal cell carcinoma, ERBB signaling pathway, WNT signaling pathway, and prostate cancer pathway. The four pathways with the strongest negative correlation were type I diabetes, primary immunodeficiency, systemic lupus erythematosus, and Alzheimer disease (Figure 6(a)). GO annotation showed five categories that were positively correlated with high levels of FLG expression: regulation of epidermis development, keratinocyte proliferation, epidermis morphogenesis, regulation of epidermal cell differentiation, and regulation of keratinocyte differentiation. GO analysis also uncovered five negatively correlated categories: cytoplasmic ubiquitin ligase complex, regulation of B cell differentiation, regulatory T cell differentiation, negative regulation of phagocytosis, and positive regulation of B cell proliferation (Figure 6(b)). These results suggest that the regulation of epidermal cell development, immune cell activation, and multiple cancer signaling pathways are critical in SKCM, which were strongly associated with FLG expression.

### 3.5. Data Validation

Using GEO database, we selected GSE15605 and GSE46517 as external data sets. There were 8 normal and 31 tumor samples in GSE46517 (*y*-axis: FLG expression; *x*-axis: groups) (Figure 7(a)) and 16 normal and 46 tumor samples in GSE15605 (*y*-axis: FLG expression; *x*-axis: groups) (Figure 7(b)). We found that FLG expression was significantly reduced in SKCM when compared the normal group (*P* < 0.01). Furthermore, immunohistochemistry analysis available from the HPA showed that in tumor tissues, FLG has lower levels of expression compared to nontumor tissues (Figures 7(c)–7(f)).

## 4. Discussion

It is well known that melanoma is highly immune-dependent malignant disease. Significant advances have been made in treating melanoma using targeted therapy and tumor immunotherapy [22]. Tumor-infiltrating immune cells (TIICs) form an ecosystem in the tumor microenvironment to regulate cancer progression and have shown potential prognostic value [23]. Besides, tumor mutational burden (TMB, mutations) has recently become an area of interest, as high TMB is associated with improved response to immune checkpoint inhibitor therapies [24]. Therefore, we selected the top 15 mutant genes from 471 melanoma patients from TCGA, and the prognosis analysis showed that only the high expression of the mutant FLG gene was significantly correlated with the poor prognosis of SKCM. The FLG protein is an important skin barrier protein; it has already been described in studies on eczema [25]. The frequency of FLG mutation in the general population is 8-10%. Approximately 10% of patients with atopic dermatitis (AD) harbor a loss-of-function mutation in the gene (FLG) that encodes filaggrin, which is important for skin barrier function [26]. However, no studies have analyzed the role of the mutant FLG in the prognosis of SKCM patients or whether it is associated with the immune microenvironment.

In our study, we found that the increased expression of FLG was significantly related to low overall survival, and its expression was significantly lower in the SKCM compared to normal tissues. This indicated that there were significant differences between FLG in normal skin tissue and melanoma tissue; FLG expression relates to several clinical characteristic including the age, tumor status, and lymph node status. Multivariate analysis showed that FLG expression is an independent prognostic factor of SKCM patient's prognosis. It is worth noting that we further analyzed the role of FLG in SKCM immune microenvironment. From TIMER, we found that lower infiltrates of B cell, CD8 + T cell, neutrophil, and dendritic cell were associated with the worse survival of SKCM patients. In latest study, Selitsky et al. highlighted the important role of B cell in modulating the antitumor immune response in SKCM [4]. Singh et al. underlined that the success of immunotherapy for melanoma appears to depend on enhancing melanoma-specific CD8+ T cell immunity since CD8+ T cells are strongly associated with direct tumor killing and a melanoma patient's survival [27]. NK cells can participate to the early immune response against melanoma and contribute to the adaptive immune response by the secretion of cytokines and by the promotion of antigen-presenting cell maturation [28]. Additionally, using CIBERSORT algorithm, we found that B cell memory, macrophage M2, and mast cell resting were apparently increased in the high expression group compared with the low expression group. These findings suggest that FLG plays a key role in the regulation and activation of SKCM immune-infiltrating cells.

What is more, we found that the expression of FLG is associated with many known cancer processes and immune response pathways. It included small cell lung cancer, basal cell carcinoma, ERBB signaling pathway, WNT signaling pathway, and prostate cancer pathway. Rha et al. highlighted that the treatment with FLG or FLA combined with paclitaxel had synergistic anticancer effects on the DLD-1 cell line [29]. More importantly, through GO enrichment analysis, FLG is closely related to epidermal cell proliferation and differentiation. Microarray revealed differential expression of several genes involved in epidermal development and keratinocyte differentiation, such as FLG, AQP9, and AKR1C3 [30]. Lippens et al. emphasized that melanoma is characterized by an imbalance towards too little apoptosis or too much cell proliferation and survival in the epidermis [31]. Kezic et al. found that epidermal filaggrin and its degradation product levels were reduced or completely lost when the FLG gene was mutated [32]. Therefore, it may be that the low expression of FLG inhibits the proliferation and differentiation of epidermal cells to achieve a good prognosis.

Although the relationship between FLG and SKCM has not been explained in detail, based on our results and previous studies on FLG, it is reasonable to believe that FLG plays a key role in the SKCM immune microenvironment. It will influence the development of the pathophysiological mechanisms of SKCM, especially the development of immune infiltration. We strongly recommend that further studies be conducted to fill in the gaps in the physiological mechanism of FLG in SKCM. Thus, FLG may be a new immune target for melanoma treatment.

## Figures and Tables

**Figure 1:** Landscape of mutation profiles in SKCM samples. Mutation information of each gene in each sample was shown in the waterfall plot, in which various colors with annotations at the bottom represented the different mutation types.

**Figure 2:** Summary of the mutation information with statistical calculations. (a–c) According to the classification of different types of mutations, missense mutations account for the largest proportion, SNP happened more frequently than insertion or deletion, and C > T was the most common of SNV. (d, e) The burden of tumor mutations in particular samples; (f) the top 10 mutated genes in SKCM; (g) the coincident and exclusive associations across mutated genes.

**Figure 3:** Survival outcome, expression difference analyzed by GEPIA, and multivariate Cox analysis of FLG: (a) differential expression of FLG in different disease state (tumor and normal); (b) survival curve of differential FLG expression; (c) differential expression of FLG in different pathological stages; (d) the expression of FLG and multivariate Cox analysis of clinicopathological factors.

**Figure 4:** Associations of FLG mutants with immune infiltration level and cumulative survival in SKCM. (a) Kaplan-Meier analysis revealed that low infiltration levels of B cell, CD8^+^ T cells, neutrophils, and dendritic cells correlated with poor survival outcomes in SKCM (*P* < 0.05). (b) Mutants of FLG conferred the low infiltration levels of immune cells.

**Figure 5:** Results of TIIC relative ratio obtained by CIBERSORT algorithm: (a) comparison of the proportion of 22 immune cells in the low and high expression groups; (b) correlation degree matrix of relative proportions of immune cells in SKCM microenvironment.

**Figure 6:** Gene function enrichment map. (a) GSEA results showed differential enrichment of genes in KEGG with FLG expression. (b) GSEA results showed differential enrichment of genes in GO with FLG expression.

**Figure 7:** Results of external data validation: (a, b) FLG expression levels in normal and SKCM tissues, as obtained from GSE46517 and GSE15605; (c–f) immunohistochemical comparison of FLG in normal skin tissues and SKCM tissues.

**Table:** (a) Association with overall survival and clinicopathologic characteristics in TCGA patients using Cox regression

Clinical characteristics	HR (95% CI)	*P* value
Age	1.02 (1.01-1.03)	0.001
Gender	1.05 (0.74-1.48)	0.794
Stage	1.57 (1.29-1.91)	0.001
FLG	1.03 (1.02-1.04)	0.001

**Table:** (b) Multivariate survival using Cox regression

Clinical characteristics	HR (95% CI)	*P* value
Age	1.01 (1.00-1.03)	0.013
Stage	0.84 (0.58-1.21)	0.355
FLG	1.19 (1.03-1.38)	0.020

**Table 2:** Gene sets enriched in phenotype.

Gene set name	NES	NOM *P* val	FDR *q* val
High expression			
KEGG_SMALL_CELL_LUNG_CANCER	1.82	0.001	0.112
KEGG_BASAL_CELL_CARCINOMA	1.72	0.002	0.194
KEGG_ERBB_SIGNALING_PATHWAY	1.65	0.016	0.280
KEGG_WNT_SIGNALING_PATHWAY	1.59	0.026	0.310
KEGG_PROSTATE_CANCER	1.51	0.042	0.355
GO_REGULATION_OF_EPIDERMIS_DEVELOPMENT	2.12	0.001	0.012
GO_KERATINOCYTE_PROLIFERATION	2.10	0.001	0.013
GO_EPIDERMIS_MORPHOGENESIS	2.07	0.001	0.014
GO_REGULATION_OF_EPIDERMAL_CELL_DIFFERENTIATION	2.04	0.001	0.015
GO_REGULATION_OF_KERATINOCYTE_DIFFERENTIATION	2.03	0.001	0.017
Low expression			
KEGG_TYPE_I_DIABETES_MELLITUS	-1.82	0.015	0.275
KEGG_PRIMARY_IMMUNODEFICIENCY	-1.75	0.017	0.095
KEGG_SYSTEMIC_LUPUS_ERYTHEMATOSUS	-1.80	0.024	0.112
KEGG_ALZHEIMERS_DISEASE	-1.61	0.032	0.118
GO_CYTOPLASMIC_UBIQUITIN_LIGASE_COMPLEX	-2.15	0.001	0.031
GO_REGULATION_OF_B_CELL_DIFFERENTIATION	-1.96	0.001	0.409
GO_REGULATORY_T_CELL_DIFFERENTIATION	-1.80	0.008	0.335
GO_NEGATIVE_REGULATION_OF_PHAGOCYTOSIS	-1.78	0.009	0.262
GO_POSITIVE_REGULATION_OF_B_CELL_PROLIFERATION	-1.80	0.011	0.330

NES: normalized enrichment score; NOM: nominal; FDR: false discovery rate.

## Data Availability

The data used to support this study is available from the first author upon request.
